RETRACTED

# The comparative effectiveness of 55 interventions in obese patients with polycystic ovary syndrome: A network meta-analysis of 101 randomized trials

**DOI:** 10.1371/journal.pone.0254412

**Published:** 2021-07-19

**Authors:** Mohamed Abdel-Maboud, Amr Menshawy, Elfatih A. Hasabo, Mohamed Ibrahim Abdelraoof, Mohamed Alshandidy, Muhammad Eid, Esraa Menshawy, Oumaima Outani, Ahmed Menshawy

**Affiliations:** 1 Faculty of Medicine, Al-Azhar University, Cairo, Egypt; 2 Faculty of Medicine, University of Khartoum, Khartoum, Sudan; 3 Faculty of Medicine, Mansoura University, Mansoura, Egypt; 4 Faculty of Medicine and Pharmacy of Rabat, Mohammed 5 University, Rabat, Morocco; 5 Department of Obstetrics and Gynecology, Faculty of Medicine, Al-Azhar University, Cairo, Egypt; Weill Cornell Medical College Qatar, QATAR

## Abstract

**Background:**

Polycystic ovary syndrome (PCOS) affects up to 18% of reproductive-age females. The prevalence of obesity in PCOS patients reaches up to 80%, which is 2-fold higher than the general population.

**Objective:**

The present study aimed to compare the effectiveness of 55 pharmacological interventions across 17 different outcomes in overweight/obese PCOS patients with hyperandrogenism manifestations for both short- and long-term follow-ups. A comprehensive literature search was performed on PubMed, Scopus, Embase, Science Direct, Web of Science, and Cochrane CENTRAL for randomized controlled trials comparing any conventional pharmacological intervention as a monotherapy or a combination in overweight/obese patients with polycystic ovary syndrome and hyperandrogenism manifestations. Extracted data included three main parameters; I. Anthropometric parameters (BMI, Waist and Hip circumferences, and Waist/HIP ratio), II. Hormonal parameters (FSH, LH, FSG, SHBG, Estradiol, Total Testosterone, Free testosterone, DHEAS, Androstenedione), and III. Metabolic parameters (Total Cholesterol, LDL-C, HDL-C, Triglycerides, Fasting glucose, Fasting glucose, HOMA-IR). Critical appraisal and risk of bias assessments were performed using the modified Jadad scale, and the overall quality of this network meta-analysis was evaluated according to the CINeMA framework. We performed both a pairwise meta-analysis and a network meta-analysis to evaluate the effect sizes with 95% CI, and we calculated the surface under the cumulative ranking curve (SUCRA) for each intervention.

**Results:**

Our final search on May 15^th^ 2021 retrieved 23,305 unique citations from searching six electronic databases. Eventually, 101 RCTs of 108 reports with a total of 8,765 patients were included in our systematic review and multi-treatments meta-analysis. 55 different interventions were included: 22 monotherapies, and 33 combinations. The two-dimensional cluster ranking of the average SUCRA values for metabolic and hormonal parameters with significant estimates revealed flutamide (77.5%, 70%; respectively) as the highest and rosiglitazone (38.2%, 26.3%; respectively) as the lowest, in terms of the overall efficacy in reducing weight and hyperandrogenism. However, cyproterone-acetate+ethinylestradiol exhibited a higher ranking in improving hormonal parameters (71.1%), but even a lower-ranking regarding metabolic parameters (34.5%).

RETRACTED

**Conclusions and relevance:**

Current evidence demonstrated the superiority of flutamide in improving both metabolic and hormonal parameters, and the higher efficacy of cyproterone-acetate+ethinylestradiol only in improving hormonal parameters. Nearly all interventions were comparable in female hormones, FGS, HDL, glucose, and insulin levels improvements.

## 1. Introduction

Polycystic ovary syndrome (PCOS) is a complex endocrinal disorder affecting up to 18% of young females [1]. The syndrome comprises of oligomenorrhea, hyperandrogenism, and polycystic findings in ovarian ultrasound [2]. While patients usually present with infertility or menstrual abnormality, they are highly susceptible to metabolic disorders such as obesity, hyperinsulinemia, and insulin resistance; thus, increasing the risks of diabetes, cardiovascular diseases, and uterine cancer -especially in overweight and obese patients [3]. For instance, the prevalence of obesity in PCOS patients reaches up to 80%, which is 2-fold higher than the general population [4].

The pathophysiology of PCOS is still unclear, but evidence suggests a mixture of environmental factors and genetic susceptibility [5]. One of the central pathogenic markers is the elevated Luteinizing Hormone (LH) levels that stimulate theca cells to produce androgens, and not enough Follicle Stimulating Hormone (FSH) to convert these androgens to estrogens [5]. Many hypotheses were presented explaining this high LH/FSH ratio including the frequent Gonadotropin-Releasing Hormone (GnRH) pulses, increased insulin resistance, and hyperinsulinemia [6].

Pharmacological interventions mainly involve: oral contraceptives, antiandrogens, oral hypoglycemics, insulin sensitizers, ovulation induction agents, and conventional obesity treatments [6]. The recently used combined oral contraceptives such as ethinylestradiol+cyproterone acetate, ethinylestradiol+desogestrel, and ethinylestradiol+drospirenone presented promising results in reducing androgen levels and regulating menstruation [7, 8].

Still, long-term use of these agents increases the risk of venous thrombosis and disrupts the metabolic parameters [9]. Hypothetically, the addition of metformin could improve glucose and lipid metabolism and reduce these severe events [10]. The problem is the required dosage of metformin can produce difficult side-effects such as nausea, diarrhea, stomach ache, and most studies measured this efficacy in the short-term [11]. On the other hand, previous pairwise meta-analyses could not address the whole range of all widely available therapies; thus, provided limited evidence to choose the most effective intervention.

RETRACTED

Given that the symptoms upon diagnosis are usually confined to irregular menstruation or infertility, physicians may disregard the possible long-term metabolic and anthropometric disturbances [6]. Subsequently, fewer studies have focused on metabolic parameters and long-term follow-up [12]. The previous studies measured limited outcomes of specific interest, leaving the final picture unclear and incomplete [13–15]. For PCOS is a chronic progressive disorder, the management should address the long-term efficacy.

Accordingly, we performed this network meta-analysis to compare the effectiveness of 55 pharmacological interventions across 17 different clinical and biochemical outcomes in overweight PCOS patients for both short- and long-term follow-ups.

## 2. Materials and methods

### 2.1 Search strategy and selection criteria

We followed the PRISMA statement guidelines (S6 File—PRISMA) [16] during the preparation of this systematic review and network meta-analysis and performed all steps in strict accordance with the Cochrane handbook of systematic reviews of intervention [17].

To synthesize the search strategy and the selected search terms, several analytical workshops, consultations of experts in the field and extensive review of the literature were employed. Eventually, a comprehensive search was employed on PubMed, Scopus, Embase, Science Direct, Web of Science, and Cochrane CENTRAL for randomized controlled trials comparing any conventional pharmacological intervention as a monotherapy or a combination in overweight/obese patients with polycystic ovary syndrome and hyperandrogenism manifestations, using relevant keywords; (Polycystic ovary syndrome [MeSH Terms]) OR (polycystic ovary syndrome[Title/Abstract])) OR (PCOS[Title/Abstract])) OR (Stein-Leventhal syndrome[MeSH Terms])) OR (Stein-Leventhal syndrome[Title/Abstract])) OR (anovulation[MeSH Terms])) OR (anovulation[Title/Abstract])) OR (amenorrhea[MeSH Terms])) OR (amenorrhea[Title/Abstract])) OR (ovarian dysfunction[Title/Abstract])) OR (ovarian failure[Title/Abstract])) OR (Oligo-amenorrhea[Title/Abstract]))) AND (metformin[Title/Abstract])) OR (metformin[MeSH Terms])) OR (liraglutide[Title/Abstract])) OR (orlistat[Title/Abstract])) OR (orlistat[MeSH Terms])) OR (inositol[MeSH Terms])) OR (inositol[Title/Abstract])) OR (oral contraceptive[MeSH Terms])) OR (oral contraceptive*[Title/Abstract])) OR (Ethinyl estradiol[MeSH Terms])) OR (Ethinyl estradiol[Title/Abstract])) OR (ethinylestradiol[MeSH Terms])) OR (ethinylestradiol[Title/Abstract])) OR (diane[Title/Abstract])) OR (cyproterone[MeSH Terms])) OR (cyproterone[Title/Abstract])) OR (combined oral contraceptive[MeSH Terms])) OR (combined oral contraceptive[Title/Abstract])) OR (OCP[Title/Abstract])) OR (CC[Title/Abstract])) OR (marvelon[MeSH Terms])) OR (marvelon[Title/Abstract])) OR (desogestrel[MeSH Terms])) OR (desogestrel[Title/Abstract])) OR (yasmin[Title/Abstract])) OR (drospirenone[Title/Abstract])) OR (letrozole[MeSH Terms])) OR (letrozole[Title/Abstract])) OR (FSH[Title/Abstract])) OR (hMG[Title/Abstract])) OR (menotropin[MeSH Terms])) OR (menotropin[Title/Abstract])) OR (pioglitazone[MeSH Terms])) OR (pioglitazone[Title/Abstract])) OR (rosiglitazone[MeSH Terms])) OR (rosiglitazone[Title/Abstract])) OR (troglitazone[MeSH Terms])) OR (troglitazone[Title/Abstract])) OR (litraglutide[Title/Abstract])) OR (flutamide[MeSH Terms])) OR (flutamide[Title/Abstract])) OR (clomiphene[MeSH Terms])) OR (clomiphene[Title/Abstract])) OR (clomifene[Title/Abstract])) OR (clomifene[MeSH Terms])) OR (chlormadinone[MeSH Terms])) OR (chlormadinone[Title/Abstract])) OR (gonadotropin[Title/Abstract])) OR (gonadotropin[MeSH Terms])) OR (simvastatin[MeSH Terms])) OR (simvastatin[Title/Abstract])) OR (atorvastatin[Title/Abstract])) OR (atorvastatin[MeSH Terms])) OR (acarbose[MeSH Terms])) OR (acarbose[Title/Abstract])) OR (alfacalcidol[Title/Abstract])) OR (anastrozole[MeSH Terms])) OR (anastrozole[Title/Abstract])) OR (clomiphene citrate[Title/Abstract])) OR (clomiphene citrate[MeSH Terms])) OR (exenatide[MeSH Terms])) OR (exenatide[Title/Abstract])) OR (folic acid[Title/Abstract])) OR (folic acid[MeSH Terms])) OR (pure follicle-stimulating hormone[MeSH Terms])) OR (pure follicle-stimulating hormone[Title/Abstract])) OR (human menopausal gonadotropins[Title/Abstract])) OR (human menopausal gonadotropins[MeSH Terms])) OR (letrozole[MeSH Terms])) OR (letrozole[Title/Abstract])) OR (liraglutide[Title/Abstract])) OR (medroxyprogesterone acetate[MeSH Terms])) OR (medroxyprogesterone acetate[Title/Abstract])) OR (N-acetyl cysteine[Title/Abstract])) OR (N-acetyl cysteine[MeSH Terms])) OR (pioglitazone[MeSH Terms])) OR (pioglitazone[Title/Abstract])) OR (rosiglitazone[Title/Abstract])) OR (rosiglitazone[MeSH Terms])) OR (sibutramine[Title/Abstract])) from inception till 28 August 2020 and search update was conducted on March 28^th^ 2021 and May 15^th^ 2021 covering all selected databases (S5 File—Search). All published articles were considered with no restriction in terms of language or date. We also searched the bibliography of included studies for additional relevant records. Metabolic parameters were not added to the final search terms due to its broader non-specific scope. Also, all variations for this broader search approach has been tested and evaluated.

RETRACTED

We included all studies satisfying the following criteria:

1. Population: overweight/obese patients (BMI more than 25 kg/m^2^) with polycystic ovary syndrome defined by Rotterdam, NIH, or Androgen Excess Society criteria for PCOs with a mutual presentation of obesity and hyperandrogenism across criteria; (2, 3) Intervention and Comparison: any conventional pharmacological intervention; (4) Outcomes: Extracted data included three main parameters; I. Anthropometric parameters (BMI, Waist and Hip circumferences, and Waist/HIP ratio), II. Hormonal parameters (FSH, LH, FSG, SHBG, Estradiol, Total Testosterone, Free testosterone, DHEAS, Androstenedione), and III. Metabolic parameters (Total Cholesterol, LDL-C, HDL-C, Triglycerides, Fasting glucose, Fasting glucose, HOMA-IR), and (5) Study design: blinded randomized controlled trials (RCTs). We excluded the following: 1) non-randomized trials, 2) open-label and cross-over studies 3) surgical, herbal, and supplemental interventions, and 4) studies whose data were unreliable for extraction and analysis including post hoc analyses and preliminary reports. Duplicates were removed and retrieved references were screened in two steps: the first step was to screen titles/abstracts for matching our inclusion criteria and the second step was to screen the full-text articles of eligible abstracts for eligibility to meta-analysis. Given the challenges in this unique design of the network-meta analysis, we included comparable RCTs in their methodology and quality to guarantee the assumption of transitivity and the lowest possible heterogeneity. We analyzed only well-designed blinded RCTs that applied globally recognized diagnostic criteria for PCOS. Regarding the BMI, we considered both the mean and the standard deviation (SD) in determining the eligibility of the studies’ population. For instance, studies that had an average BMI above 25 but had a standard deviation that crosses the 25-mean into a lower value for some patients were excluded. Also, we separated studies with short-term follow-ups from those with long-term follow-ups in the statistical combinations. Eventually, each included intervention was administered as primary therapy in its original study. So, a critical distinction has to be made between a tertiary/off-label use of a drug and the primary use of the same drug.

RETRACTED

It is worth mentioning that PCOS can present differently in the clinical practice that is infertility, anovulation, irregular menses, hyperandrogenism, or metabolic disturbances. Accordingly, when comparing 55 interventions, it is clear that each group of these therapies is usually administered to only address a part of the problem (i.e. Clomiphene citrate for ovulation, Rosiglitazone for insulin resistance, etc.), so it would not be fair to compare these agents to each other regarding the same outcome. With that in mind, we had two prospects when planning for this study. Firstly, we could have focused the study on the used interventions a particular PCOS phenotype (irregular menses, insulin resistance, hyperlipidemia, etc.) only. Even though this option would have been much simpler to handle, the work would have contributed more to widening the current knowledge gap. Given that PCOS has a progressive nature, it does not restrain itself to the presented phenotype, let alone that the borders that should determine different managements between various phenotypes are inevitably interleaving -implying a dire need for a much comprehensive investigation. Alternatively, we selected 17 measurable parameters that are mutual between various phenotypes and grouped them into anthropometric, metabolic, and hormonal parameters. Following, we examined the effect of each intervention on each parameter of these 17 parameters (whether this intervention is usually used to address this parameter or not, such as Clomiphene citrate effect on LDL). That is how even when intervention X has primary use for the first five parameters (with a secondary or tertiary effect on the rest) and intervention Y has primary use for the last five parameters (with secondary or tertiary effect on the rest), we can still draw an overall performance across parameters between the two interventions in an objective manner. Eventually, the data of this extensive analysis would help in drawing step-wise management for different phenotypes based on the best performing intervention across the prioritized parameters of that phenotype (such as hormonal parameters in irregular menses presentation, and metabolic-anthropometric parameters in morbid obesity presentation, and all hormonal-metabolic-anthropometric parameters in multiple severe presentations). This algorithm will further promote the clinical practice to be more data-driven instead of theory-driven regarding PCOS management.

Eight independent authors extracted the relevant data from the included studies, four authors (M.A.M., A.M., E.A.H., and M.I.A) performed the literature search and validation, then, another four authors (M.A., M.E., E.M., and O.O.) re-performed the search and validation. Disagreements were resolved through discussion and consensus among the reviewers. The screening and de-duplication were conducted through Endnote X7 and Microsoft Excel 2016. The extracted data included the following:

1. Baseline characteristics (Study ID, Year, Country, Intervention groups, Dosage, Sample size, Age in years, blinding, Diagnostic criteria, Follow up duration in weeks, and Resistance)
2. Study outcomes: I. Anthropometric parameters, II. Hormonal, and III. Metabolic parameters -as previously defined.

RETRACTED

Critical appraisal and risk of bias assessments of the included RCTs were performed using the modified Jadad scale from Oxford University [18]. This eight-item scale was designed to evaluate randomization, blinding, dropouts, criteria of inclusion and exclusion, adverse effects, and statistical analysis (S1 File; S1 Table in S1 File). The score ranges from 0 (the lowest quality) to 8 (the highest quality). Articles with scores of 4–8 indicate good to excellent quality, while those with 0–3 denote poor to low quality. The overall quality of this network meta-analysis was evaluated according to the CINeMA framework. Funnel plots were constructed to make visual assessments of possible publication bias.

### 2.2 Data analysis

Statistical analyses were performed using Stata 16.0 software. First, we conducted a pair-wise meta-analysis employing the IVhet random-effects model. All reported units were converted to standard SI units. All data were continuous (means and standard deviations "SD") and were pooled as weighted mean differences (MD) with 95% confidence intervals. Missing SD was calculated from the standard error or 95% CI or range according to Wan et al. [19] or obtained from SD of baseline and SD of change according to Cochrane 16.1.3.2 [17]. Heterogeneity between trials was examined visually and statistically through Chi-square and I2 tests: values of 0%-40%, 30%-60%, 50%-90%, and 75%-100% represented low, moderate, substantial, and considerable heterogeneity; respectively. P<0.1 was set as a level of significant heterogeneity, according to Cochrane Handbook recommendations. When considerable heterogeneity was detected, we conducted a sensitivity analysis to determine the source of heterogeneity by excluding one study at a time.

Second, a network meta-analysis was performed with a frequentist framework to compare different interventions that have no direct comparisons. We applied the node-splitting and loop-specific approaches to verify inconsistencies across the network, where a p<0.05 indicated a significant inconsistency. When no significant inconsistency was detected, we employed a consistency model; otherwise, an inconsistency model was adopted. We also utilized a global inconsistency test based on a random-effects design-by-treatment interaction model. Additionally, the surface under the curve ranking area (SUCRA) was calculated to rank different interventions for each outcome. Further, a meta-regression was conducted to examine the relationship between anthropometric, hormonal, and metabolic parameters.

RETRACTED

## 3. Results

### 3.1 Characteristics and quality of included studies

Our updated search retrieved 23,305 unique citations from searching electronic databases. Following title and abstract screening, 408 full-text articles were retrieved and screened for eligibility. Of them, 307 articles were excluded, and 101 RCTs [20–32, 33, 34–43, 44, 45–54, 55, 56–65, 66, 67–76, 77, 78–87, 88, 89–98, 99, 100–109, 110, 111–120] (108 reports) (n = 8,765 patients) were reviewed in detail and included in this multi-treatment meta-analysis (PRISMA flow diagram; Fig 1). The updated search identified 16 new study [121–128, 129–136], however, they could not be added to our analysis due to the following causes: five studies failed to meet our BMI criteria [136–126], three studies included irrelevant interventions [133–135], two studies had an open-label design [127, 128], two studies measured different outcomes [131, 132], one study had a cost-effectiveness design [121], one study had a post-hoc design [129], one study had no treatment control [122], and one study included pregnant patients [130]. Additionally, the bibliography of the included RCTs was manually searched, but no further records were added. All of the included studies were performed between 1987 and 2020; 37 studies in Europe, 32 studies in the Middle East, 20 studies in North America, 8 studies in Asia, and 4 studies in South America.

**Fig 1:** A PRISMA flow diagram illustrates the search results, de-duplication, screening and the selection process.

55 different interventions were included: 22 monotherapies, and 33 combinations. The monotherapies included acarbose (ACR), alfacalcidol (ALF), anastrozole (ANZ), clomiphene citrate (CC), exenatide (EXN), folic acid (FA), flutamide (FLT) pure follicle-stimulating hormone (FSH), human menopausal gonadotropins (HMG), inositol (INS), letrozole (LET), liraglutide (LIR), metformin (MET), medroxyprogesterone acetate (MPA), N-acetyl cysteine (NAC), orlistat (ORL), pioglitazone (PGZ), placebo (PLC), rosiglitazone (RGZ), sibutramine (SBT), simvastatin (SMV), and troglitazone (TGZ).

RETRACTED

The combinations included acarbose+clomiphene citrate (ACR+CC), alfacalcidiol+metformin (ALF+MET), atorvastatin+metformin (ATR+MET), bromocriptine+clomiphene citrate (BRM+CC), bromocriptine+metformin (BRM+MET), clomiphene citrate+dexamethasone (CC+DEX), clomiphene citrate+ketoconazole (CC+KTZ), clomiphene citrate+l-carnitine (CC+LC), clomiphene citrate+l-carnitine+metformin (CC+LC+MET), clomiphene citrate+metformin (CC+MET), clomiphene citrate+N-acetylcysteine (CC+NAC), clomiphene citrate+rosiglitazone (CC+RGZ), chlormadinone acetate+ethinylestradiol (CHA+EE), cyproterone acetate+ethinylestradiol (CPA+EE), cyproterone acetate+ethinylestradiol+metformin (CPA+EE+MET), cyproterone acetate+ethinylestradiol+metformin+orlistat (CPA+EE+MET+ORL), cyproterone acetate+ethinylestradiol+orlistat (CPA+EE+ORL), cyproterone acetate+ethinylestradiol+spironolactone (CPA+EE+SPR), dexamethasone+metformin (DEX+MET), desogestrel+ethinylestradiol (DGT+EE), drospirenone+ethinylestradiol (DPN+EE), drospirenone+ethinylestradiol+metformin (DPN+EE+MET), ethinylestradiol+flutamide+levonorgestrel (EE+FLT+LVT), ethinylestradiol+gestodene (EE+GTN), ethinylestradiol+metformin+norgestimate (EE+MET+NRG), ethinylestradiol+norgestimate (EE+NRG), folic acid+inositol (FA+INS), flutamide+metformin (FLT+MET), human menopausal gonadotropins+ leuprolide (HMG+LPR), inositol+monacolin k (INS+MNK), letrozole+metformin (LET+MET), metformin+rosuvastatin (MET+RSV), and metformin+simvastatin (MET+SMV).

A network map was formed to visually display the size of studies involved in each direct comparison for each outcome (Fig 2), and a summary table was drawn to detail each included study (Table 1). We divided comparisons of the same treatment into two categories based on the follow-up duration, where studies below 24 weeks grouped as a short and intermediate-term, and those from 24 weeks onward grouped as a long term. The mark (#) at the end of a treatment’s abbreviation indicates a short term follow up.

**Fig 2:** Network graphs of eligible comparisons for efficacy. The size of the circles is proportional to sample size, and the width of lines is proportional to the number of trials. Interventions: acarbose (ACR), alfacalcidol (ALF), anastrozole (ANZ), clomiphene citrate (CC), exenatide (EXN), folic acid (FA), flutamide (FLT) pure follicle-stimulating hormone (FSH), human menopausal gonadotropins (HMG), inositol (INS), letrozole (LET), liraglutide (LIR), metformin (MET), medroxyprogesterone acetate (MPA), N-acetyl cysteine (NAC), orlistat (ORL), pioglitazone (PGZ), placebo (PLC), rosiglitazone (RGZ), sibutramine (SBT), simvastatin (SMV), and troglitazone (TGZ). Acarbose+clomiphene citrate (ACR+CC), alfacalcidiol+metformin (ALF+MET), atorvastatin+metformin (ATR+MET), bromocriptine+clomiphene citrate (BRM+CC), bromocriptine+metformin (BRM+MET), clomiphene citrate+dexamethasone (CC+DEX), clomiphene citrate+ketoconazole (CC+KTZ), clomiphene citrate+l-carnitine (CC+LC), clomiphene citrate+l-carnitine+metformin (CC+LC+MET), clomiphene citrate+metformin (CC+MET), clomiphene citrate+N-acetylcysteine (CC+NAC), clomiphene citrate+rosiglitazone (CC+RGZ), chlormadinone acetate+ethinylestradiol (CHA+EE), cyproterone acetate+ethinylestradiol (CPA+EE), cyproterone acetate+ethinylestradiol+metformin (CPA+EE+MET), cyproterone acetate+ethinylestradiol+metformin+orlistat (CPA+EE+MET+ORL), cyproterone acetate+ethinylestradiol+orlistat (CPA+EE+ORL), cyproterone acetate+ethinylestradiol+spironolactone (CPA+EE+SPR), dexamethasone+metformin (DEX+MET), desogestrel+ethinylestradiol (DGT+EE), drospirenone+ethinylestradiol (DPN+EE), drospirenone+ethinylestradiol+metformin (DPN+EE+MET), ethinylestradiol+flutamide+levonorgestrel (EE+FLT+LVT), ethinylestradiol+gestodene (EE+GTN), ethinylestradiol+metformin+norgestimate (EE+MET+NRG), ethinylestradiol+norgestimate (EE+NRG), folic acid+inositol (FA+INS), flutamide+metformin (FLT+MET), human menopausal gonadotropins+ leuprolide (HMG+LPR), inositol+monacolin k (INS+MNK), letrozole+metformin (LET+MET), metformin+rosuvastatin (MET+RSV), and metformin+simvastatin (MET+SMV).

RETRACTED

**Table 1:** Shows baseline and summary data of patients in included studies.

Author	Year	Country	Groups	Dosage	Sample Size	Age	Blinding	Diagnostic Criteria	Folllow Up (Weeks)	Resistance	Author	Year	Country	Groups	Dosage	Sample Size	Age	Blinding	Diagnostic Criteria	Folllow Up (Weeks)	Resistance
						Mean ± SD (years)											Mean ± SD (years)				
**Azziz et al,**	2003	United States	PLC		73	29.3 ± 5.6	Double	NIH Criteria	20	NA	**Azziz et al,**	2001	United States	PLC		73	30.1 ± 6.0	Double	NIH Criteria	44	NA
			TGZ	150 mg/day	78	29.3 ± 5.6								TGZ	150 mg/day	78	28.9 ± 5.4				
			TGZ	300 mg/day	77	29.3 ± 5.6								TGZ	300 mg/day	77	29.2 ± 5.8				
			TGZ	600 mg/day	77	29.3 ± 5.6								TGZ	600 mg/day	78	29.0 ± 5.2				
**Aroda et al,**	2009	United States	PLC		10	27.0 ± 1.0*	Single	NIH Criteria	24	NA	**Hassan et al, (a)**	2001	Egypt	CC+KTZ	100 mg/day+400 mg/day	25	NA	Single	NIH Criteria	36	NA
			PGZ	45 mg/day	13	28.0 ± 1.0*								CC	100 mg/day	38	NA				
**Hassan et al, (b)**	2001	Egypt	CC+KTZ	100 mg/day+400 mg/day	12	NA	Single	NIH Criteria	36	CC	**Abu Hashim et al,**	2010	Egypt	LET	2.5 mg/day	123	28.3 ± 2.7	Single	Rotterdam Criteria	8	CC
			CC	100 mg/day	5	NA								CC+MET	150 mg/day+500 mg tid	127	26.2 ± 2.2				
**Bridger et al,**	2006	Canada	MET	750 mg bid	11	16.07 ± 0.97	Double	NIH Criteria	12	NA	**Brettenthaler et al,**	2004	United Kingdom	PGZ	30 mg/day	17	30.2 ± 1.4*	Double	NIH Criteria	12	NA
			PLC		11	16.08 ± 1.39								PLC		18	30.6 ± 1.1*				
**Bilgir et al,**	2009	Turkey	CPA+EE	2 mg/day+35 μg/day	20	24.3 ± 5.7	Single	Rotterdam Criteria	12	NA	**Bhattacharya et al, (24 wks)**	2012	India	DGT+EE	0.15 mg/day+0.03 mg/day	58	22.24 ± 4.47	Double	Androgen Excess Society criteria	24	NA
														CPA+EE	2 mg/day+0.03 mg/day	56	22.32 ± 4.17				
			CPA+EE+MET	2 mg/day+35 μg/day+1700 mg/day	20	25.2 ± 4.6								DPN+EE	3 mg/day+0.03 mg/day	57	22.33 ± 4.76				
**Bhattacharya et al, (48 wks)**	2012	India	DGT+EE	0.15 mg/day+0.03 mg/day	58	22.24 ± 4.47	Double	Androgen Excess Society criteria	48	NA	**Benelli et al,**	2016	Italy	FA+INS^1^+ INS^2^	200 μg bid+550 mg bid+13.8 mg bid	21	23 ± 6.8	Single	Rotterdam Criteria	24	NA
			CPA+EE	2 mg/day+0.03 mg/day	56	22.32 ± 4.17															
			DPN+EE	3 mg/day+0.03 mg/day	57	22.33 ± 4.76								FA	200 μg bid	25	25 ± 7.3				
**Badawy et al, (a)**	2009	Egypt	ANZ	1 mg/day	115	23.8 ± 3.1*	Single	Rotterdam Criteria	10	NA	**Badawy et al, (b)**	2009	Egypt	LET	5 mg/day	218	27.1 ± 3.2*	Single	Rotterdam Criteria	10	NA
			CC	100 mg/day	101	25.3 ± 2.9*								CC	100 mg/day	220	29.3 ± 2.9*				
**Badawy et al,**	2008	Egypt	CC	100 mg/day	160	24.1 ± 3.1*	Single	Rotterdam Criteria	16	CC	**Chou et al,**	2003	Brazil	MET	500 mg tid	14	24 ± 5	Double	NIH Criteria	12	NA
			HMG	75 IU/day	158	26.3 ± 3.0*								PLC		16	24.5 ± 6.1				
**Celik et al,**	2012	Turkey	MET	2000 mg/day	20	25.9 ± 5.7	Single	Rotterdam Criteria	12	NA	**Cakiroglu et al,**	2013	Turkey	DPN+EE	30 μg/day+3 mg/day	10	NA	Single	Rotterdam Criteria	24	NA
			MET+RSV	2000 mg/day+10 mg/day	20	27.6 ± 5.9								DPN+EE+MET	850 mg/day+30 μg/day+3 mg/day	9	NA				
**Dravecká et al,**	2016	Slovakia	ALF	1 μg/day	9	29.33 ± 4.89	Single	Androgen Excess Society criteria	24	NA	**Dodson et al,**	1987	United States	HMG	300 IU	6	31.92	Single	NIH Criteria	4	CC
			ALF+MET	1 μg/day+1700–2550 mg/day	11	29.2 ± 5.42															
			MET	1700–2550 mg/day	12	27.6 ± 4.96								HMG+LPR	300 IU + 1mg	7	31.92				
**De leo et al,**	2010	Italy	DPN+EE	3 mg/day+30 μg/day	10	16 to 35	Single	Rotterdam Criteria	12	NA	**Davar et al,**	2011	Iran	CC+MET	100 mg/day+1500 mg/day	50	29.55 ± 3.47	Single	Rotterdam Criteria	8	CC
			CHA+EE	2 mg/day+30 μg/day	10	16 to 35															
			EE+GTN	75 μg/day+30 μg/day	10	16 to 35								LET+MET	5 mg/day+1500 mg/day	48	28.54 ± 3.13				
			DGT+EE	150 μg/day+30 μg/day	10	16 to 35															
**Essah et al,**	2011	United States	EE+MET+NRG	0.035 mg+500 mg+0.25 mg tid	10	NA	Double	Rotterdam Criteria	12	NA	**Elnashar et al,**	2006	Egypt	CC+DEX	100 mg/day+2 mg/day	40	23.38 ± 3.5941	Double	Rotterdam Criteria	8	CC
			EE+NRG+PLC	0.035 mg+0.25 mg	9	NA								CC+PLC	100 mg/day	40	25.15 ± 2.3783				
**El-khayat et al,**	2016	Egypt	CC	100 mg/day	50	26.58 ± 2.93	Double	Rotterdam Criteria	24	CC	**El Sharkwy et al, (a)**	2019	Egypt	CC+LC+MET	150 mg/day+3 g/day+850–1700 mg/day	138	25.7 ± 1.7	Double	Rotterdam Criteria	12	CC
			LET	5 mg/day	50	25.82 ± 3.62								CC+MET+PLC	150 mg/day+850–1700 mg/day	136	26.1 ± 2.2				
**El Sharkwy et al, (b)**	2019	Egypt	CC+NAC	150 mg/day+600 mg tid	82	26.6 ± 1.5	Double	Rotterdam Criteria	12	CC	**Fuxotta et al,**	2010	Argentina	MET	1500 mg/day	14	25.47 ± 4.82	Double	Androgen Excess Society criteria	16	NA
			CC+LC	150 mg/day+3 g/day	80	26.2 ± 2.8								PLC		15	24.7 ± 3.46				
**Fruzzetti et al,**	2017	Italy	MET	1500 mg/day	22	22.3 ± 6.0	Single	Rotterdam Criteria	24	NA	**Frøssing et al,**	2018	Denmark	LIR	1.8 mg/day	44	NA	Double	Rotterdam Criteria	26	NA
			INS^1^	4 g/day	24	21.6 ± 6.6								PLC		21	NA				
**Fleming et al,**	2002	United Kingdom	MET	850 mg bid	45	28.6 (26.9–30.3)**	Double	NIH Criteria	14	NA	**Figurová et al,**	2017	Slovakia	MET	1700–2550 mg/day	12	27.6 ± 4.96	Single	Androgen Excess Society criteria	24	NA
			PLC		47	29.2 (27.5–30.7)**								ALF	1 μg/day	9	29.33 ± 4.89				
														ALF+MET	1 μg/day+1700–2550 mg/day	11	29.2 ± 5.42				
**Feng et al,**	2016	China	CPA+EE+MET	2 mg/day+35 μg/day+425–850 mg bid	41	27.86 ± 3.79	Double	Rotterdam Criteria	12	NA	**Gupta et al,**	2016	United States	PGZ	45 mg/day	16	29.68 ± 1.10*	Double	NIH Criteria	24	NA
			CPA+EE	2 mg/day+35 μg/day	41	28.57 ± 3.04								PLC		16	30.56 ± 1.08*				
**Glintborg et al,**	2006–2009	Denmark	PGZ	30 mg/day	15	32 (26–36)***	Double	NIH Criteria	16	NA	**Gerli et al,**	2003	Italy	INS^1^	100 mg bid	136	28.6 (26.9–30.3)**	Double	Rotterdam Criteria	1	NA
			PLC		15	34 (29–38)***								PLC		147	29.2 (27.5–30.7)**				
**Genazzani et al,**	2008	Italy	FA+INS^1^	200 μg/day+2 g/day	10	NA	Single	Rotterdam Criteria	12	NA	**Gambineri et al, (24 wks)**	2004–2006	Italy	PLC		19	26.0 ± 5.0	Single	Rotterdam Criteria	24	NA
														MET	850 mg bid	20	28.0 ± 8.0				
			FA	200 μg/day	10	NA								FLT	250 mg bid	17	26.0 ± 6.0				
														FLT+MET	250 mg bid+850 mg bid	20	26.0 ± 5.0				
**Gambineri et al, (48 wks)**	2006	Italy	PLC		19	26.0 ± 5.0	Single	Rotterdam Criteria	48	NA	**Gadir et al,**	1991	United Kingdom	HMG	150 IU	30	26.5 ± 0.73*	Single	Rotterdam Criteria	20	CC
			MET	850 mg bid	20	28.0 ± 8.0															
			FLT	250 mg bid	17	26.0 ± 6.0								FSH	75 IU	29	27.3 ± 0.66*				
			FLT+MET	250 mg bid+850 mg bid	20	26.0 ± 5.0															
**Hutchison et al,**	2008	Australia	MET	1000 mg bid	19	34.1	Single	NIH Criteria	24	NA	**Hoeger et al, (a)**	2008	United States	MET	1700 mg/day	10	16.0 ± 1.7	Double	NIH Criteria	24	NA
														PLC		11	15.4 ± 1.7				
			CPA+EE	2 mg/day+35 μg/day	19	34.1															
														DGT+EE	0.15 mg/day+30 μg/day	11	15.4 ± 1.4				
**Hoeger et al, (b)**	2008	United States	DPN+EE+MET	3 mg/day+30 μg/day+2000 mg/day	18	14.7 ± 1.6	Double	NIH Criteria	24	NA	**Hanjalic-beck et al,**	2010	Germany	MET	2550 mg/day	19	28.0	Double	NIH Criteria	12	NA
			DPN+EE+PLC	3 mg/day+30 μg/day	18	15.8 ± 1.6								ACR	300 mg/day	18	28.0				
**Jakubowicz et al,**	2001	United States	MET	500 mg tid	26	27.0 ± 1.0*	Double	NIH Criteria	4	NA	**Jamilian et al, (a)**	2017	Iran	MET	500 mg tid	30	25.9±4.8	Double	Rotterdam Criteria	12	NA
			PLC		22	27 .0 ± 1.0*								FA+INS^1^	200 μg bid+2 g bid	30	27.7±5.2				
**Jamilian et al, (b)**	2018	Iran	MET	500 mg tid	30	27.7 ± 3.4	Double	Rotterdam Criteria	12	NA	**Javanmanesh et al,**	2016	United Kingdom	MET	500 mg tid	48	29.75 ± 4.90	Double	Rotterdam Criteria	24	NA
			FA+INS^1^	200 μg bid+2 g bid	30	28.5 ± 4.7								NAC	600 mg tid	46	28.98 ± 4.42				
**Jensterle et al,**	2008	Slovenia	MET	850 mg bid	15	23.1 ± 3.7	Single	NIH criteria	24	NA	**Kumar et al,**	2014	India	MET	500 mg tid	30	NA	Single	Rotterdam Criteria	12	NA
			RGZ	4 mg/day	11	25.0 ± 4.9								ORL	120 mg bid	30	NA				
**Koiou et al,**	2013	Greece	SBT	10 mg qd	28	25.7 ± 5.9	Single	Rotterdam Criteria	24	NA	**Kocak et al,**	2002	Turkey	CC+MET	100 mg/day+850 mg bid	28	26.2 ± 3.7	Double	NIH Criteria	8	CC
			ORL	120 mg bid	22	25.7 ± 5.9								CC+PLC	100 mg/day	28	27.1 ± 4.5				
**Kjøtrød et al,**	2009	Norway	MET	2000 mg/day	17	28.9 (26.7–31.0)**	Double	Rotterdam Criteria	14	NA	**Kilic et al,**	2011	Turkey	MET	850 mg bid	24	28.7 ± 3.7	Double	Rotterdam Criteria	24	NA
			PLC		19	29.9 (28.1–31.8)**								DGT+EE	0.15 mg/day+0.03 mg/day	25	29.0 ± 3.5				
**Khorram et al,**	2006	United States	CC+MET	100 mg/day+500 mg tid	16	28.4 ± 0.78*	Single	Rotterdam Criteria	3	NA	**Kebapcilar et al,**	2010	Turkey	CPA+EE	2 mg/day+35 μg/day	12	23.2 ± 5.1	Single	Rotterdam Criteria	12	NA
														CPA+EE+MET	2 mg/day+35 μg/day+850 mg bid	12	24.9 ± 4.8				
			CC	100 mg/day	15	28.0 ± 1.1*								MET	850 mg bid	12	24.4 ± 6.2				
														CPA+EE+SPR	2 mg/day+35 μg/day+100 mg/day	12	23.4 ± 5.8				
**Kebapcilar et al,**	2009	Turkey	CPA+EE	2 mg/day+35 μg/day	22	24.1 ± 5.6	Single	Rotterdam Criteria	12	NA	**Kazerooni et al,**	2010	United States	MET+SMV	500 mg tid+20 mg/day	42	25.6 ± 4.32	Double	Rotterdam Criteria	12	NA
			CPA+EE+MET	2 mg/day+35 μg/day+1700 mg/day	21	25.1 ± 1.4								MET+PLC	500 mg tid	42	24.9 ± 5.81				
**Kazerooni et al,**	2009	United States	CC+MET	100 mg/day+500 mg tid	20	24.5 ± 5.16	Double	Rotterdam Criteria	4	CC	**Kaya et al,**	2015	Turkey	DPN+EE	3 mg/day+3 μg/day	25	23.0 ± 5.0	Double	Rotterdam Criteria	24	NA
			CC+PLC	100 mg/day	20	25.47 ± 4.7								DPN+EE+MET	3 mg/day+3 μg/day+850 mg bid	25	24.0 ± 4.0				
**Kaya et al,**	2012	Turkey	DPN+EE	3 mg/day+3 μg/day	19	23.2 ± 5.4	Double	Androgen Excess Society criteria	24	NA	**Karimzadeh et al,**	2007	Iran	MET	500 mg tid	100	27.2 ± 6.8	Double	Rotterdam Criteria	12	NA
			DPN+EE+MET	3 mg/day+3 μg/day+850 mg bid	18	23.0 ± 4.5								PLC		100	28.6 ± 7.4				
**Ko et al,**	2001			500 mg tid			Single	NIH Criteria			**Lord et al,**	2006	United Kingdom	MET	500 mg tid	21	27.76 ± 4.89	Double	Rotterdam Criteria	12	NA
														PLC		19	30.63 ± 4.84				
**De Leo et al,**	2013	Italy	INS^1^+MNK	1.5 g/day+3 g bid	20	24 to 32	Single	Rotterdam Criteria	24	NA	**Lemay et al,**	2006	Canada	RGZ	4 mg/day	10	26.8 ± 5.7	Single	Rotterdam Criteria	24	NA
			INS^1^	1.5 g/day	20	24 to 32															
														CPA+EE	2 mg/day+35 μg/day	7	20.0 ± 1.5				
			MET	850 mg bid	20	24 to 32															
**Legro et al,**	2014	United States	CC	50 mg/day	376	28.8 ± 4.0	Double	Rotterdam Criteria	16	NA	**Legro et al,**	2007	United States	CC+PLC	50 mg/day	209	27.9 ± 4.0	Double	NIH criteria and Rotterdam diagnostic criteria	24	NA
														MET+PLC	500 mg tid	208	28.1 ± 4.0				
			LET	2.5 mg/day	374	28.9 ± 4.5															
														CC+MET	50 mg/day+500 mg tid	209	28.3 ± 4.0				
**Ladson et al,**	2011	United States	MET	500 mg bid			Double	NIH Criteria	24	NA	**Morin-Papunen et al,**	2000	Finland	MET	1000 mg bid	16	29.9 ± 1.5*	Single	NIH Criteria	24	NA
			PLC		59	28.8 ± 4.6								CPA+EE	2 mg/day+35 μg/day	16	28.8 ± 1.0*				
**Moini et al,**	2015	Iran	ORL	120 mg tid	50	26.8 ± 5.16	Double	Rotterdam Criteria	12	NA	**Mohsen et al,**	2012	Egypt	CC+RGZ	100 mg+4 mg bid	46	25.9 ± 2.7	Single	Rotterdam Criteria	12	NA
			PLC		50	27.42 ± 3.31								CC	100 mg/day	45	26.4 ± 2.9				
**Mohiyideen et al,**	2013	United Kingdom	RGZ	4 mg od	18	29.0 ± 1.0	Double	Rotterdam Criteria	12	NA	**Moghetti et al,**	2000	Italy	MET	500 mg tid	12	23.9 ± 1.2*	Double	NIH Criteria	24	NA
			MET	500 mg bid	17	30.0 ± 0.9								PLC		11	21.4 ± 1.4*				
**Mehrabian et al,**	2016	Iran	MET	1000 mg/day	37	29.18 ± 8.288	Single	NIH Criteria	24	NA	**Machado et al,**	2012	Brazil	MET	850 mg bid	21	27.4 ± 3.8	Double	Rotterdam Criteria	8	NA
			EE+FLT+LVT	0.03 mg/day +62.5 mg/day+0.15 mg/day	37	29.0 ± 7.663															
														PLC		15	28.2 ± 3.2				
			SMV	20 mg/day	37	29.15 ± 8.261															
**Nylander et al,**	2017	Denmark	LIR	1.8 mg/day	48	31.4 (24.6–35.6)***	Double	Rotterdam Criteria	26	NA	**Nestler et al,**	1999	United States	INS^2^	1200 mg/day	22	29.0 ± 6.0	Double	NIH Criteria	6 to 8	NA
			PLC		24	26.2 (24.8–31.5)***								PLC		22	26.0 ± 5.0				
**Nestler et al,**	1998	United States	MET	500 mg tid	35	29.0 ± 1.0*	Single	NIH Criteria	5	NA	**Nordio et al,**	2012	Italy	INS^1^	550 mg bid	24	28.2 ± 1.5	Single	Rotterdam Criteria	24	NA
			PLC		26	28.0 ± 1.0*								INS^1^+INS^2^	550 mg bid+13.8 mg bid	26	27.9 ± 1.4				
**Onalan et al, (a)**	2005	Turkey	MET	500–850 mg bid	10	24.6 ± 4.8	Double	NIH Criteria	24	NA	**Onalan et al, (b)**	2005	Turkey	MET	500–850 mg bid	10	31.8 ± 4.0	Double	NIH Criteria	24	NA
			PLC		9	27.3 ± 4.4								PLC		8	21.2 ± 5.5				
**Pasquali et al, (4 wks)**	2000	Italy	MET	850 mg bid	12	31.6 ± 10.3	Double	NIH Criteria	4	NA	**Pasquali et al, (28 wks)**	2000	Italy	MET	850 mg bid	20	31.6 ± 10.3	Double	NIH Criteria	28	NA
			PLC		8	36.3 ± 9.5								PLC		20	36.3 ± 9.5				
**Parsanezhad et al, (12 wks)**	2004	Iran	BRM+CC	7.5 mg/day+150 mg/day	47	25.02 ± 2.7	Double	NIH Criteria	12	CC	**Parsanezhad et al, (24 wks)**	2004	Iran	BRM+CC	7.5 mg/day+150 mg/day	47	25.02 ± 2.7	Double	NIH Criteria	24	CC
			CC+PLC	150 mg/day	53	24.87 ± 2.9								CC+PLC	150 mg/day	53	24.87 ± 2.9				
**Parsanezhad et al,**	2002	Iran	CC+DEX	200 mg/day+2 mg/day	20	23.56	Double	NIH Criteria	3	CC	**Rautio et al, (12 wks)**	2005	Finland	MET	500–1000 mg bid	16	29.6 ± 1.1*	Single	Rotterdam Criteria	12	NA
			CC+PLC	200 mg/day	20	23.36								CPA+EE	2 mg+0.035 mg	16	29.6 ± 1.1*				
**Rautio et al, (24 wks)**	2005	Finland	MET		16	29.6 ± 1.1*	Single	Rotterdam Criteria	24	NA	**Rautio et al,**	2006	Finland	RGZ	4–8 mg/day	15	26.7 ± 1.1*	Double	Rotterdam Criteria	16	NA
			CPA+EE		16	29.6 ± 1.1*								PLC		15	30.1 ± 2.1*				
**Rautio et al,**	2007	Finland	RGZ	4–8 mg/day	12	29.1 ± 1.2*	Double	Rotterdam Criteria	16	NA	**Rouzi et al,**	2006	Saudi Arabia	CC+RGZ	100 mg/day+4 mg bid	12	28.58 ± 3.73	Single	NIH Criteria	12	CC
			PLC		14	29.1 ± 1.2*								CC+MET	100 mg/day+500 mg tid	13	27.38 ± 4.29				
**Sova et al,**	2013	Finland	MET	1000 mg bid	23	29.2 ± 4.6	Double	Rotterdam Criteria	12	NA	**Sönmez et al,**	2005	Turkey	ACR+CC	300 mg/day+100 mg/day	15	26.13 ± 5.08	Double	NIH Criteria	12	CC
			PLC		27	27.4 ± 4.9								CC+MET	100 mg/day+1700 mg/day	15	26.0 ± 3.92				
**Song et al,**	2018	China	CPA+EE+ORL	2 mg/day+35 μg/day+120 mg tid	60	26.77 ± 4.12	Double	Rotterdam Criteria	12	NA	**Sathyapalan et al,**	2010	United Kingdom	ATR+MET	20 mg/day+500 mg tid	19	26.6 ± 1.2*	Double	NIH Criteria	24	NA
			CPA+EE+MET	2 mg/day+35 μg/day+500–1500 mg/day	60	28.63 ± 5.12															
			CPA+EE+MET+ORL	2 mg/day+35 μg/day+500–1500 mg/day+120 mg tid	60	27.57 ± 4.58								MET+PLC	500 mg tid	18	28.8 ± 1.8*				
			CPA+EE	2 mg/day+35 μg/day	60	27.68 ± 4.99															
**Tfayli et al,**	2011	United States	DPN+EE	3 mg/day+30 μg/day	20	16.2 ± 0.3*	Double	NIH Criteria	24	NA	**Tang et al,**	2006	United Kingdom	MET	850 mg bid	69	29.7 ± 3.7	Double	Rotterdam Criteria	24	NA
			RGZ	4 mg/day	17	15.7 ± 0.3*								PLC		74	29.8 ± 3.8				
**Villaseca et al,**	2004	Chile	MPA	10 mg/day	15	23.9 ± 5.1	Single	NIH Criteria	12	NA	**Vanky et al, (a)**	2004	Norway	MET+PLC	850 mg tid	15	28.3 ± 5.0	Double	Rotterdam Criteria	8	NA
														BRM+MET	5 mg/day+850 mg tid	14	28.3 ± 5.0				
			CPA+EE	2 mg/day+35 μg/day	16	22.4 ± 6.1															
														DEX+MET	0.5 mg/day+850 mg tid	12	28.3 ± 5.0				
**Vanky et al, (b) (8 wks)**	2004	Norway	DEX+MET	0.5 mg/day+850 mg tid	18	26.4 ± 3.8	Double	Rotterdam Criteria	8	NA	**Vanky et al, (b) (26 wks)**	2004	Norway	DEX+MET	0.5 mg/day+850 mg tid	18	26.4 ± 3.8	Double	Rotterdam Criteria	26	NA
			MET+PLC	850 mg tid	20	30.6 ± 5.9								MET+PLC	850 mg tid	20	30.6 ± 5.9				
**Vandermolen et al,**	2001	United States	MET	500 mg tid	11	29.0 ± 1.2*	Double	NIH Criteria	7	CC	**Van Santbrink et al,**	2005	The Netherlands	MET	850 mg bid	11	28.0 (22–32)****	Double	NIH Criteria	5	NA
			PLC		14	30.0 ± 1.0*								PLC		9	28.0 (24–34)****				
**Wu et al,**	2008	China	CPA+EE	2 mg/day+35 μg/day	7	25.0 ± 4.3	Double	Rotterdam Criteria	12	NA	**Yarali et al,**	2002	Turkey	MET	850 mg bid	16	29.7 ± 5.6	Double	NIH Criteria	6	CC
			MET	500 mg tid	7	25.6 ± 3.6															
														PLC		16	28.4 ± 5.1				
			CPA+EE+MET	2 mg/day+35 μg/day+500 mg tid	6	24.5 ± 2.4															
**Yilmaz et al,**	2005	Turkey	MET	850 mg bid	43	24.67 ± 4.6	Single	Rotterdam Criteria	24	NA	**Zheng et al,**	2019	China	EXN	10 μg bid	31	27.2 ± 1.76*	Single	Rotterdam Criteria	12	NA
			RGZ	4 mg/day	45	25.13 ± 4.43								MET	1000 mg bid	32	27.7 ± 1.64*				

INS^1^: Myo-Inositol; INS^2^: D-Chiro-Inositol

*: Mean SEM

**:Mean (Confidence intervals 95%)

***:median (25%–75% quartiles)

****: Median (Range)

Interventions: acarbose (ACR), alfacalcidol (ALF), anastrozole (ANZ), clomiphene citrate (CC), exenatide (EXN), folic acid (FA), flutamide (FLT) pure follicle-stimulating hormone (FSH), human menopausal gonadotropins (HMG), inositol (INS), letrozole (LET), liraglutide (LIR), metformin (MET), medroxyprogesterone acetate (MPA), N-acetyl cysteine (NAC), orlistat (ORL), pioglitazone (PGZ), placebo (PLC), rosiglitazone (RGZ), sibutramine (SBT), simvastatin (SMV), and troglitazone (TGZ). Acarbose+clomiphene citrate (ACR+CC), alfacalcidiol+metformin (ALF+MET), atorvastatin+metformin (ATR+MET), bromocriptine+clomiphene citrate (BRM+CC), bromocriptine+metformin (BRM+MET), clomiphene citrate+dexamethasone (CC+DEX), clomiphene citrate+ketoconazole (CC+KTZ), clomiphene citrate+l-carnitine (CC+LC), clomiphene citrate+l-carnitine+metformin (CC+LC+MET), clomiphene citrate+metformin (CC+MET), clomiphene citrate+N-acetylcysteine (CC+NAC), clomiphene citrate+rosiglitazone (CC+RGZ), chlormadinone acetate+ethinylestradiol (CHA+EE), cyproterone acetate+ethinylestradiol (CPA+EE), cyproterone acetate+ethinylestradiol+metformin (CPA+EE+MET), cyproterone acetate+ethinylestradiol+metformin+orlistat (CPA+EE+MET+ORL), cyproterone acetate+ethinylestradiol+orlistat (CPA+EE+ORL), cyproterone acetate+ethinylestradiol+spironolactone (CPA+EE+SPR), dexamethasone+metformin (DEX+MET), desogestrel+ethinylestradiol (DGT+EE), drospirenone+ethinylestradiol (DPN+EE), drospirenone+ethinylestradiol+metformin (DPN+EE+MET), ethinylestradiol+flutamide+levonorgestrel (EE+FLT+LVT), ethinylestradiol+gestodene (EE+GTN), ethinylestradiol+metformin+norgestimate (EE+MET+NRG), ethinylestradiol+norgestimate (EE+NRG), folic acid+inositol (FA+INS), flutamide+metformin (FLT+MET), human menopausal gonadotropins+ leuprolide (HMG+LPR), inositol+monacolin k (INS+MNK), letrozole+metformin (LET+MET), metformin+rosuvastatin (MET+RSV), and metformin+simvastatin (MET+SMV).

RETRACTED

All of the included studies were randomized, blinded, and were treated as an intention to treat (ITT) analysis; thus, exhibiting a low risk of bias. The funnel plot was visually symmetrical (S1 File; S1 Fig in S1 File), indicating no possible publication bias, and the further Egger’s test revealed no small study effect (P = 0.35). The overall quality of evidence for each outcome in this network meta-analysis was evaluated according to the CINeMA framework, revealing high-quality evidence (S3 File—CINeMA). Overall, 692 direct comparisons and 7,166 indirect comparisons were obtained for the 17 outcomes from 101 trials.

### 3.2 Pairwise meta-analyses

We performed a pairwise meta-analysis for RCTs that compared the same interventions employing the random-effects IVhet model. The results of these analyses are displayed in S4 File—Pairwise plots. No statistically significant difference was observed among interventions regarding WHR (I^2 = 0%, P = 0.986), FSH (I^2 = 0%, P = 1.000), Estradiol (I^2 = 0%, P = 1.000), FGS (I^2 = 0%, P = 0.991), Free Testosterone (I^2 = 0%, P = 1.000), and HDL (I^2 = 0%, P = 0.896). Pooled analyses were homogenous

For BMI, only the following comparisons revealed significance: CPA+EE+MET+ORL# vs. CPA+EE# (MD = −3.2, 95% CI [−6.3, −0.1]), CPA+EE+MET+ORL# vs. CPA+EE+ORL# (MD = −5, 95% CI [−8.4, −1.6]), FLT vs. MET (MD = −4, 95% CI [−6.6, −1.3]), FLT vs. PLC (MD = −4.95, 95% CI [−7.6, −2.2]), and FLT+MET vs. PLC (MD = −3.4, 95% CI [−6.3, −0.6]). Pooled analysis was homogenous (I^2 = 34.29%, P = 0.013).

RETRACTED

For LH *(mIU/ml)*, only the following comparisons revealed significance: MET vs. PLC (MD = −4.5, 95% CI [−8.3, −0.8]). LIR was inferior to PLC in reducing LH levels (MD = 23.9, 95% CI [18.2, 29.5]). Pooled analysis was moderately heterogeneous (I^2 = 65.27%, P< 0.001), and heterogeneity did not resolve after further sensitivity analysis.

For SHBG *(nmol/L)*, only the following comparisons revealed significance: CPA+EE vs. MET (MD = 113.7, 95% CI [84.5, 142.9]), CPA+EE vs. RGZ (MD = 89, 95% CI [51, 127]), DGT+EE vs. PLC (MD = 103, 95% CI [65.6, 140.3]), DPN+EE vs. DGT+EE (MD = 33.2, 95% CI [3.3, 63.1]), DPN+EE vs. RGZ (MD = 97, 95% CI [60.4, 133.5]), and INS+MNK vs. INS (MD = 46, 95% CI [1.42, 90.5]). Pooled analysis was moderately heterogeneous (I^2 = 76.33%, P< 0.001), and heterogeneity did not resolve after further sensitivity analysis.

For Total Testosterone *(ng/dl)*, only the following comparisons revealed significance: CPA+EE vs. MET (MD = −21.3, 95% CI [−40.1, −2.4]), DGT+EE vs. MET (MD = −29, 95% CI [−52.5, −5.4]), DGT+EE vs. PLC (MD = −30.6, 95% CI [−55.8, −5.4]), and CC+DEX# vs. PLC (MD = −51, 95% CI [−93.5, −8.4]). Pooled analysis was homogenous (I^2 = 0%, P = 0.541).

For DHEAS *(μg/dl)*, only the following comparisons revealed significance: FLT vs. MET (MD = −74.6, 95% CI [−127.7, −21.4]), FLT vs. PLC (MD = −69.8, 95% CI [−125, −14.7]), INS# vs. PLC (MD = −147, 95% CI [−255.6, −38.3]), and MET+RSV# vs. MET# (MD = −121.3, 95% CI [−237.3, −5.2]). Pooled analysis was homogenous (I^2 = 22.23%, P = 0.104).

For Total Cholesterol *(mg/dl)*, only the following comparisons revealed significance: MET+SMV# vs. MET# (MD = −53.2, 95% CI [−97.1, −9.4]). Pooled analysis was homogenous (I^2 = 0%, P = 0.991).

For LDL *(mg/dl)*, only the following comparisons revealed significance: INS+MNK vs. INS (MD = −77.9, 95% CI [−103.5, −52.2]), INS+MNK vs. MET (MD = −71, 95% CI [−92.6, −49.3]), MET vs. DGT+EE (MD = −30.3, 95% CI [−59.4, −1.2]), MET# vs. PLC (MD = −10.3, 95% CI [−18.4, −2.3]), MET+SMV# vs. MET# (MD = −21, 95% CI [−0.8, −41.2]), and ORL# vs. PLC (MD = −28.4, 95% CI [−44.6, −12.2]). Pooled analysis was moderately heterogeneous (I^2 = 70.17%, P< 0.001), and heterogeneity did not resolve after further sensitivity analysis.

For Triglycerides *(mg/dl)*, only the following comparisons revealed significance: FLT vs. MET (MD = −27.5, 95% CI [−53.1, −1.9]), FLT vs. PLC (MD = −32.7, 95% CI [−6.5, −58.9]), and MET+RSV# vs. MET# (MD = −41.5, 95% CI [−77.6, −5.3]). DPN+EE was inferior to RGZ in reducing Triglycerides levels (MD = 84.2, 95% CI [51.4, 117.1]). Pooled analysis was homogenous (I^2 = 39.13%, P = 0.003).

RETRACTED

For Fasting Glucose *(mg/dl)*, only the following comparisons revealed significance: MET# vs. PLC (MD = −5.4, 95% CI [−10.1, −0.7]), and MET# vs. ORL# (MD = −21.6, 95% CI [−33.3, −9.9]. ORL# was inferior to PLC in reducing Fasting Glucose levels (MD = 16.1, 95% CI [4.8, 27.5]). Pooled analysis was homogenous (I^2 = 0%, P = 0.698).

For Fasting Insulin *(pmol/L)*, only the following comparisons revealed significance: CC+MET vs. CC (MD = −279.1, 95% CI [−352.9, −205.4]), and MET vs. CC (MD = −250.7, 95% CI [−324.4, −176.9]). CPA+EE and DPN+EE were inferior to RGZ in reducing Fasting Insulin levels (MD = 63.648, 95% CI [4.4, 122.8]) and (MD = 62.6, 95% CI [5.7, 119.5]); respectively. Pooled analysis was moderately heterogeneous (I^2 = 61.7%, P< 0.001), and heterogeneity did not resolve after further sensitivity analysis.

For HOMA-IR, only the following comparisons revealed significance: ALF vs. ALF+MET (MD = −1.1, 95% CI [−2.2, −0.04]), CC+MET vs. CC (MD = −1.9, 95% CI [−2.7, −1]), CPA+EE+MET# vs. CPA+EE# (MD = −0.6, 95% CI [−1.1, −0.09]), DGT+EE vs. CPA+EE (MD = −1.1, 95% CI [−1.7, −0.4]), DGT+EE vs. DPN+EE (MD = −1.1, 95% CI [−1.7, −0.5]), MET vs. ALF+MET (MD = −1.9, 95% CI [−3, −0.9]), MET vs. CC (MD = −1.1, 95% CI [−1.9, −0.2]), MET vs. CPA+EE (MD = −1.3, 95% CI [−2.5, −0.2]), PGZ vs. PLC (MD = −2.1, 95% CI [−3, −1.1]), and RGZ vs. CPA+EE (MD = −1.4, 95% CI [−2.7, −0.1]). Pooled analysis was moderately heterogeneous (I^2 = 68.32%, P< 0.001), and heterogeneity did not resolve after further sensitivity analysis.

### 3.3 Network meta-analyses

Additionally, we performed a frequentist network meta-analysis. Following the results of node-splitting analyses, we adopted the consistency model. The estimated value of between-study variance in the network ranged from 2.2 to 309.7. Among indirect comparisons, significant inconsistencies were identified in the closed-loop of MET#-ORL#-PLC and DGT+EE-DPN+EE-MET-RGZ (S1 File; S2 Fig in S1 File). Further, employing the Global test based on the random-effects design-by-treatment interaction model, χ2 values ranged from 0.1 (1 df.) to 10.6 (12 df.), P-value: 0.2–0.5; respectively. Moreover, comparisons with significant heterogeneity or incoherence were downgraded (S3 File—CINeMA).

Results of each direct and indirect comparison in the network meta-analysis are detailed extensively in S2 File—NMA League Tables. In addition to the significant estimates of the pairwise meta-analysis, the following comparisons revealed a statistical significance as well. Compared with placebo, MET+RSV# and CPA+EE+SPR# were superior at reducing LDL levels (MD = -29.1, 95% CI [-51.9, -93.7]) and (MD = -25.3, 95% CI [-48.2, -2.5]); respectively, DPN+EE+MET was inferior at reducing Triglycerides levels (MD = 83.6, 95% CI [16.8, 150.4]), and CC was inferior at reducing Fasting Insulin levels (MD = 254.9, 95% CI [176.4, 333.4]) (Fig 3).

RETRACTED

**Fig 3:** Forest plots show the mean difference (MD) of different interventions compared with placebo for each outcome, along with the associated 95% CI. Interventions: acarbose (ACR), alfacalcidol (ALF), anastrozole (ANZ), clomiphene citrate (CC), exenatide (EXN), folic acid (FA), flutamide (FLT) pure follicle-stimulating hormone (FSH), human menopausal gonadotropins (HMG), inositol (INS), letrozole (LET), liraglutide (LIR), metformin (MET), medroxyprogesterone acetate (MPA), N-acetyl cysteine (NAC), orlistat (ORL), pioglitazone (PGZ), placebo (PLC), rosiglitazone (RGZ), sibutramine (SBT), simvastatin (SMV), and troglitazone (TGZ). Acarbose+clomiphene citrate (ACR+CC), alfacalcidiol+metformin (ALF+MET), atorvastatin+metformin (ATR+MET), bromocriptine+clomiphene citrate (BRM+CC), bromocriptine+metformin (BRM+MET), clomiphene citrate+dexamethasone (CC+DEX), clomiphene citrate+ketoconazole (CC+KTZ), clomiphene citrate+l-carnitine (CC+LC), clomiphene citrate+l-carnitine+metformin (CC+LC+MET), clomiphene citrate+metformin (CC+MET), clomiphene citrate+N-acetylcysteine (CC+NAC), clomiphene citrate+rosiglitazone (CC+RGZ), chlormadinone acetate+ethinylestradiol (CHA+EE), cyproterone acetate+ethinylestradiol (CPA+EE), cyproterone acetate+ethinylestradiol+metformin (CPA+EE+MET), cyproterone acetate+ethinylestradiol+metformin+orlistat (CPA+EE+MET+ORL), cyproterone acetate+ethinylestradiol+orlistat (CPA+EE+ORL), cyproterone acetate+ethinylestradiol+spironolactone (CPA+EE+SPR), dexamethasone+metformin (DEX+MET), desogestrel+ethinylestradiol (DGT+EE), drospirenone+ethinylestradiol (DPN+EE), drospirenone+ethinylestradiol+metformin (DPN+EE+MET), ethinylestradiol+flutamide+levonorgestrel (EE+FLT+LVT), ethinylestradiol+gestodene (EE+GTN), ethinylestradiol+metformin+norgestimate (EE+MET+NRG), ethinylestradiol+norgestimate (EE+NRG), folic acid+inositol (FA+INS), flutamide+metformin (FLT+MET), human menopausal gonadotropins+ leuprolide (HMG+LPR), inositol+monacolin k (INS+MNK), letrozole+metformin (LET+MET), metformin+rosuvastatin (MET+RSV), and metformin+simvastatin (MET+SMV).

The ranking probabilities of the highest and lowest intervention for each outcome are available in S1 File; S3 Fig in S1 File. The two-dimensional cluster ranking of the average SUCRA values for metabolic and hormonal parameters with significant estimates revealed FLT (77.5%, 70%; respectively) as the highest and RGZ# (38.2%, 26.3%; respectively) as the lowest, in terms of the overall efficacy. However, CPA+EE exhibited a higher ranking in improving hormonal parameters (71.1%), but even a lower-ranking regarding metabolic parameters (34.5%) (Fig 4).

RETRACTED

**Fig 4:** A rankogram show the cumulative ranking of the average SUCRA values for each intervention across all metabolic and hormonal parameters.

### 3.4 Meta-regressions

We further employed multiple regression models to assess the interaction between anthropometric, metabolic, and hormonal parameters with significant estimates. The results of these meta-regressions are available in S1 File; S4 Fig in S1 File. Changes in BMI were significantly associated with changes in SHBG (Coefficient 0.012; P = 0.000, R2 = 51.6%), Total Testosterone (Coefficient -0.031; P = 0.000, R2 = 34%), and DHEAS (Coefficient 0.004; P = 0.02, R2 = 8%). The inversed regression for the effect of BMI on these parameters had a lower R2 value for SHBG (2.62%) Total Testosterone (0%), and DHEAS (0%).

In contrast, LDL and Triglyceride levels showed no significant associations with Total Testosterone (P = 0.86, P = 0.54; respectively) or DHEAS levels (P = 0.31, P = 0.76; respectively). However, changes in LDL and Triglyceride levels were significantly associated with changes in SHBG (Coefficient 0.012; P = 0.001, R2 = 7.8%) and (Coefficient 0.225; P = 0.000, R2 = 16.4%); respectively. The inversed regression for the effect of LDL and Triglycerides on SHBG was not significant (P = 0.43, P = 0.53; respectively). Likewise, no significant associations were detected between HOMA-IR and either SHBG (P = 0.9) or Total Testosterone (P = 0.95) or DHEAS (P = 0.97).

## 4. Discussion

In the present systematic review and network meta-analysis: 55 interventions were evaluated for efficacy in reducing weight and hyperandrogenism through 7,858 comparisons across 17 outcomes. The included interventions can be categorized pharmacologically into ten categories: Oral contraceptives, Gonadotropins modulators, Estrogen modulators, Aromatase inhibitors, Catecholamines modulators, Antiandrogens, Antidiabetics, Cholesterol modulators, Antioxidants, and Anti-inflammatories. After a long chain of analyses, the competition settled between Antiandrogens, Oral contraceptives, Anti-diabetics, Cholesterol modulators, and combinations in-between categories.

Flutamide, an antiandrogen, proved efficacy in improving anthropometric, androgenic, and lipid parameters. Cyproterone acetate+ethinylestradiol, an antiandrogen with an oral contraceptive, demonstrated the highest efficacy in improving androgenic parameters. However, it did not exhibit any superiority in the remaining parameters. Inositol+monacolin K, an antidiabetic and a cholesterol modulator, displayed efficacy in improving androgenic and lipid parameters. Likewise, metformin+simvastatin/rosuvastatin and orlistat, an antidiabetic and cholesterol modulators, significantly improved lipid parameters. Nonetheless, these improvements were only observable in the short term follow-up.

RETRACTED

Ideally, all interventions were comparable in female hormones, FGS, HDL, glucose, and insulin levels improvements. As an exception, liraglutide, an antidiabetic, showed a significantly lower efficacy in reducing LH levels. Clomiphene citrate, an estrogen modulator, was the least effective agent in improving insulin levels. Eventually, pioglitazone, an antidiabetic, demonstrated efficacy in reducing HOMA-IR.

Meanwhile, results of meta-regression revealed no significant associations between changes in hormonal and metabolic parameters. Even those few significant associations had a very small R-squared. This finding indicates that a drug’s action on hormonal parameters does not necessarily modify metabolic parameters and vice versa. Also, this finding is counter-intuitive to previous studies that attributed PCOS progression to lipid metabolism disturbance [137, 138]. This implication may provide further justification for the combined therapies of different categories. However, our analysis revealed that most combinations were not promising. For instance, the combinations of flutamide+metformin, ethinylestradiol+flutamide+levonorgestrel, cyproterone acetate+ethinylestradiol+metformin, and cyproterone acetate+ethinylestradiol+orlistat were inferior to either agent separately. Still, it remains questionable whether a future combination of flutamide+cyproterone acetate+ethinylestradiol can create better potentials.

On the other hand, meta-regression revealed a significant effect of hormonal parameters on anthropometric parameters. This finding could explain why traditional obesity interventions show limited efficacy and limited duration in obese PCOS patients [139, 140]. Further, it implies that: when treating PCOS obesity, physicians should consider interventions with hormonal adjustments such as flutamide.

Given the high prevalence of obesity among PCOS patients, effective treatments that improve both obesity and reproductive functions are urgently needed [141, 142]. Evidence indicates that PCOS patients with overweight/obesity show a higher risk of long-term morbidity including anovulation, diabetes, and cardiovascular disorders. The cumulative ranking of flutamide as the best intervention across outcomes has many implications [143, 144].

Flutamide works by inhibiting androgen uptake or nuclear binding in the target tissues [145]. However, it has extensive metabolism, leaving only 2.5% of its concentration in plasma one hour after intake [146]. This critical issue generates an urgent need for a modified preparation. Otherwise, the ultimate current solution is multiple fractionated doses, which raises concerns about cost-effectiveness. It is important to point out that the best and worst treatment can potentially alternate according to clinical judgments. For instance, most PCOS patients are diagnosed because of irregular menstruation or infertility; however, an additional presentation with obesity, insulin resistance, hirsutism, and acne requires further consideration. Patients’ value of whether they desire pregnancy or not changes the main course of management.

RETRACTED

The mainstream literature approaches PCOS either as a mere metabolic disturbance or a fertility challenge [147–150]. Furthermore, meta-analyses are highly selective to certain outcomes of interest as ovulation, pregnancy, metabolic syndrome, and weight loss. These attitudes, for sure, serves the value of many patients but simultaneously ignores the value of another considerable group of patients. Those patients may not be interested in pregnancy nor having serious weight problems; rather, they want their body to function with normal feminine biology for their sexual, social, and psychological lives. Likewise, previous network meta-analyses included a limited number of outcomes and interventions of particular categories and either presented no significant results or a low to very low evidence. These limitations mainly due to the inclusion of poorly designed RCTs, the limited outcomes, the limited comparisons, the incomprehensive literature search, the inclusion of post hoc analyses, and the unreliable statistical combinations.

In our systematic review and network meta-analysis: we assessed multi-dimensional outcomes, developed strict inclusion criteria, separated short-term from long term comparisons, and analyzed only well-designed RCTs in the past 30 years. Our findings settle a group of assumptions and advocate a reliable reference for future clinical decisions and guidelines. To the best of our knowledge: this is the first meta-analysis to investigate this size of outcomes with this number of interventions in the management of PCOS. The findings for various treatments involved were consistent for all measured outcomes, and the evidence presented was highly rated.

Even so, some limitations can be identified in our work: most RCTs had relatively small sample sizes; thus, the wide 95% CI of most comparisons indicates insufficient power. Also, we restricted the average BMI to over 25; hence, the implications can only apply to overweight/obese PCOS patients. The modifications in the clinical definitions and diagnostic criteria of PCOS may contribute to the clinical heterogeneity.

RETRACTED

Overall, the current evidence demonstrated the superiority of flutamide in improving both metabolic and hormonal parameters. And the higher efficacy of cyproterone acetate+ethinylestradiol only in improving hormonal parameters. Nearly all interventions were comparable in female hormones, FGS, HDL, glucose, and insulin levels improvements. Even though inositol+monacolin K, metformin+simvastatin/rosuvastatin, and orlistat ranked higher in improving lipid parameters, their efficacy lasted only for short-term follow-ups. Liraglutide exhibited the lowest efficacy in reducing LH levels, and clomiphene citrate was the least effective agent in improving insulin levels. Pioglitazone demonstrated the highest efficacy in reducing HOMA-IR on the long-term follow-up. In the management of PCOS: a drug’s action on hormonal parameters does not necessarily modify metabolic parameters and vice versa. Obesity in PCOS is a unique case of obesity that should not be merely addressed by traditional weight-loss interventions. Prospective large-scale clinical trials are crucially required to study the appropriate dosage of flutamide and to assess the efficacy of combined flutamide+cyproterone acetate+ethinylestradiol.

## Supporting information

S1 File (DOCX)

S2 File Displays extended NMA League Tables. (XLSX)

S3 File Contains CINeMA frameworks for each outcome. (XLSX)

S4 File Shows the forest plots of the pairwise meta-analyses. (PDF)

S5 File Contains the detailed search terms for each database. (DOCX)

S6 File The NMA PRISMA Checklist. (DOCX)
